RETRACTED

# Application Effect of Robot-Assisted Laparoscopy in Hepatectomy for Colorectal Cancer Patients with Liver Metastases

**DOI:** 10.1155/2022/5492943

**Published:** 2022-06-16

**Authors:** Shiguang Li, Linxi Fu

**Affiliations:** ^1^Medical Department of Wuhan Ninth Hospital, Wuhan, Hubei 430080, China; ^2^Public Health Department, Honggangcheng Street Community Health Service Center, Qingshan District, Wuhan, Hubei 430080, China

## Abstract

**Objective:**

Application effect of Leonardo's robot-assisted laparoscopy in hepatectomy for colorectal cancer patients with liver metastases.

**Methods:**

A total of 122 patients with sCRLM treated in our hospital from May 2015 to June 2018 were selected and divided into observation group (*n* = 61) and control group (*n* = 61) according to random number table method. The observation group was treated with robot-assisted laparoscopic hepatectomy, while the control group was treated with conventional laparoscopic hepatectomy. The perioperative time, intraoperative blood transfusion, intraoperative blood loss, average intraoperative blood transfusion, and hepatic portal occlusion time of the two groups were observed. Serum cortisol (Cor), norepinephrine (NE), and glucose (Glu) levels were detected before and after surgery in the two groups. The oxygen consumption and carbon dioxide output of patients were measured 1 day before surgery and 1~3 days after surgery, and the resting energy expenditure (REE) value was calculated. The levels of CD3+, CD4+, and CD8+ were determined by flow cytometry. The incidence of complications was compared between the two groups. Patients were followed up for 3 years after discharge, and Kaplan-Meier method was used to analyze the survival of the two groups.

**Results:**

The operation time, intraoperative blood transfusion, intraoperative blood loss, and average intraoperative blood transfusion in the observation group were all less than those in the control group, and the differences were statistically significant (*P* < 0.05). Three days after operation, the levels of serum Cor, NE, and Glu were increased in both groups, and the observation group was lower than the control group; the difference was statistically significant (*P* < 0.05). The REE level of observation group was lower than that of control group after 1 day, 2 days, and 3 days after surgery, and the difference was statistically significant (*P* < 0.05). Three days after operation, the levels of serum CD3+ and CD4+ were decreased in both groups, and the observation group was higher than the control group; the difference was statistically significant (*P* < 0.05). The incidence of complications in the observation group (3.28%) was lower than that in the control group (13.11%); the difference was statistically significant (*P* < 0.05).There was no significant difference in survival rate between the two groups after 1, 2, and 3 years of follow-up (*P* > 0.05).

RETRACTED

**Conclusion:**

The application of robot-assisted laparoscopy in patients with sCRLM can effectively improve the perioperative situation of patients, reduce stress, energy metabolism, and immune damage, and reduce the incidence of complications.

## 1. Introduction

Colorectal cancer is a common malignant tumor disease in China, and about 60% of patients can develop liver metastases, and about 2/3 of patients with synchronous colorectal liver metastases (sCRLM) may die [1, 2]. Hepatectomy should be performed on patients who meet the surgical indications for hepatectomy. Liver is the largest solid organ of the human body, with special anatomical structure and complex physiological functions. Laparoscopic hepatectomy has high risks. With the development of medical technology, laparoscopic and robotic surgery are more and more widely used in surgical operation, and minimally invasive surgery has the advantages of less trauma and quick recovery [3–5]. Compared with laparoscopy, Da Vinci robotic surgery has better operability and stability [6–8]. As an intelligent surgical platform, Leonardo's robot surgical system has a three-dimensional stereoscopic field of view and a mechanical wrist with 7 degrees of freedom, has the advantages of fine anatomy and precise anastomosis, and is helpful for laparoscopic hepatectomy. Surgical injury can trigger stress response of the body, lead to a series of neuroendocrine changes, activate the sympathetic-adrenal medulla axis and the hypothalamic-pituitary-adrenal cortex axis, which can increase the level of catecholamines and glucocorticoids in the blood, and change the body's metabolism and internal environment. sCRLM is a consumptive disease. Traumatic surgery can change the basal metabolic rate and internal environment of the patient and make the patient's body in a high metabolic state, resulting in postoperative recovery difficulties. According to relevant reports, the stability of surgical microenvironment is closely related to the success rate of surgery [9, 10]. The purpose of this study was to explore the effects of robot-assisted laparoscopy on energy metabolism and long-term prognosis of patients with sCRLM.

## 2. Materials and Methods

### 2.1. General Information

A total of 122 patients with sCRLM treated in our hospital from May 2015 to June 2018 were selected and divided into observation group and control group according to the random number table method, with 61 cases in each group. All patients participating in this clinical study were fully informed about this study and signed the informed consent. This study was approved by the hospital ethics committee, and the patients' informed consent was ensured under the supervision of the ethics committee.

RETRACTED

### 2.2. Inclusion Criteria

These include the following: ① patients with sCRLM confirmed by clinicopathological diagnosis; ② all patients were treated with radical resection of colorectal cancer, and no tumor residue was found; ③ no large blood vessel infiltration, hepatic vein, or portal vein tumor thrombus was found by imaging examination; ④ Child-Pugh liver function class was A or B; ⑤ no severe organ dysfunction was observed; ⑥ all patients volunteered to participate in this study.

### 2.3. Exclusion Criteria

These include the following: ① patients with unresectable extrahepatic metastases; ② patients with other malignant tumors; ③ patients with incomplete clinicopathological data; ④ patients with extensive infiltration of adhesion between the tumor and the surrounding tissue; ⑤ patients with severe obesity, severe infection, intestinal perforation, and massive intestinal gas accumulation, or acute intestinal obstruction; and ⑥ pregnant and lactating patients.

### 2.4. Methods

The observation group was treated with robot-assisted laparoscopic hepatectomy, while the control group was treated with laparoscopic hepatectomy. Before surgery, the patient's past medical history and present medical history as well as the results of routine examinations should be fully understood. For the observation group, Leonardo's robot was prepared. Leonardo's robot system was a mobile platform and a three-dimensional imaging video image platform composed of the master console operated by surgeons, the instrument arm, the endoscope arm, and the surgical instruments. Before the operation, the integrity of each system was carefully checked, the link of each part was completed, the machine was opened 30 minutes in advance, and the robot was debugged to make it in the standby state. According to the habits of the chief surgeon, the ultrasonic knife, laparoscopic hepatic resection instrument, bipolar electrode coagulation forceps, endoscopic cutting closure device, and nonabsorbable titanium clamp were prepared. The special instruments for robot surgery include ultrasonic knife core, long-hole bipolar electrocoagulation grasping forceps, special needle holder, and ultrasonic knife sheath. The initial position of the patient was supine. After combined general anesthesia with endotracheal intubation and intravenous anesthesia, an operation hole was established, and the Trocar was placed according to the location and size of the lesion and the body shape of the patient. A No. 11 blade was used to make an arc incision along the upper edge of the umbilicus, and a pneumoperitoneum needle was used to establish a CO_2_ pneumoperitoneum. The pneumoperitoneum was 12-14 mmHg (1 mmHg = 0.133 kPa). The 12 mm Trocar was connected to the lens arm, and the camera lens was placed. A Trocar with a diameter of 8 mm was placed at the anterior axillary line 2~4 cm below the left costal margin and connected with the mechanical arm I. A Trocar with a diameter of 8 mm was placed at the midclavicular line 2~4 cm below the right costal margin and connected with the robotic arm II, and an ultrasonic knife and bipolar electric coagulation forceps were placed. An 8 mm Trocar was placed at the right axillary midline, and a 12 mm Trocar was placed at the midclavicular line 2~4 cm below the left umbilicus as an assistant approach. According to the surgical requirements, the mechanical arm III was connected to the right axillary midline, and the grasping forceps was placed. For patients requiring endoscopic biliary tract exploration, a 12 mm Trocar was placed under the xiphoid process and a choledochoscope was placed. In order to avoid the collision of the robotic arms, the operation holes should be arc-distributed centered on the surgical target area with a spacing of 5-6 cm. During the operation, the scope of the lesion and the plane of liver were determined by a sterile endoscopic B-ultrasound probe. The robotic instrument arm and lens arm were separated from the corresponding Trocar. The patient was placed in a secondary position, i.e., high head and low foot, with the operating table at a 30° angle to the horizontal position, and the hepatoduodenal ligament was exposed. The self-made first hepatic portal occlusion device was preset to expose and separate the perihepatic ligament. In nonanatomic hepatectomy, the first hepatic porta was not treated. In anatomic hepatectomy, the first hepatic porta was dissected, and the hepatic artery and the left branch of portal vein on the affected side were separated, ligated, and severed, respectively, and the liver parenchyma was severed with ultrasonic scalpel and bipolar coagulation forceps. The blood vessels and biliary duct with diameter ≤ 5 mm in the liver were clipped with successive titanium clips and then cut off. The hepatic vein, larger branches of hepatic vein, bile duct, and Glisson sheath were cut off with a linear cutter and clipped and then sutured and ligated for reinforcement. If there was intrahepatic duct bleeding, No. 4-0 vascular line was used for suture and ligature. When the liver parenchyma was severed, if there was serious bleeding in the liver resection surface, the first hepatic porta should be blocked to block the blood flow into the liver, and bipolar electric coagulation forceps should be used to stop the bleeding, and then, the liver tumor was excised with an ultrasonic scalpel. Finally, the specimen was removed, and the liver resection surface and abdominal cavity were washed. If no biliary leakage or bleeding was found, the abdominal drainage tube was placed and the operating table was restored to a horizontal position before the abdominal cavity was closed until the end of the operation. In the control group, the entire abdominal and pelvic cavity was explored by laparoscopy to determine the resectability of the liver metastases. After the blood vessels were severed and the bowel was dissociated, the bowel distal to the tumor was cut off, and the stapler nail seat was inserted. Finally, the intestinal tube was put back into the abdominal cavity, the incision under the costal margin was closed, and the intestinal anastomosis was completed under laparoscopy. Finally, the drainage tube was placed in the surgical incision.

RETRACTED

### 2.5. Observation Indicators

These include the following: ① baseline data. ② Clinical manifestations of patient surgery during the perioperative period include the operation time, intraoperative blood transfusion, intraoperative blood loss, average intraoperative blood transfusion, and hepatic porta occlusion time were observed in the two groups. ③ Stress response indicators include cortisol (Cor), norepinephrine (NE), and glucose (Glu). The above indexes were determined by enzyme-linked immunosorbent assay. Blood samples were taken from the patient's fasting cubital venous blood (5 ml each time, centrifuged at 3000 r/min for 10 min at 4°C, and the supernatant was stored at -80°C). ④ Energy metabolism was measured by the oxygen consumption and carbon dioxide production of patients 1 day before surgery and 1-3 days after surgery (at 6 am before getting up). The value of resting energy expenditure (REE) was calculated by computer based on indirect calorimetry theory. ⑤ The evaluation index of immune function is CD3+, CD4+, and CD8+ levels. The above indicators were measured by flow cytometry. ⑥ Complications were observed. ⑦ Survival curve analysis was calculated by Kaplan-Meier method. Follow-up methods include telephone and outpatient service. The frequency of follow-up was once/month in the first year, once/3 months in the second year, and once/6 months in the third year.

### 2.6. Statistical Methods

The SPSS 20.0 statistical software was used to analyze and process the data, and the measurement data were expressed as *x̅*±*s*. Independent sample *t* test was used for intergroup comparison, and paired *t* test was used for intragroup comparison before and after treatment. Count data were expressed as frequency and composition ratio. Disordered classification data were compared using *χ*^2^ test or Fisher's exact probability test. *P* < 0.05 indicated that the difference was statistically significant.

RETRACTED

## 3. Results

### 3.1. Comparison of Baseline Data between the Two Groups

There were no statistically significant differences in baseline data such as gender and age between the two groups, indicated that the two groups of patients were comparable (see Table 1).

### 3.2. Comparison of Perioperative Conditions between the Two Groups

The operation time, intraoperative blood transfusion, intraoperative blood loss, and average intraoperative blood transfusion in the observation group were all less than those in the control group, and the differences were statistically significant (*P* < 0.05) (see Table 2).

### 3.3. Comparison of Stress Response Index Levels between the Two Groups before and after Surgery

Before operation, there was no significant difference in the levels of serum Cor, NE, and Glu between the two groups (*P* > 0.05). Three days after operation, the levels of serum Cor, NE, and Glu in both groups were increased, and the observation group was lower than the control group; the difference was statistically significant (*P* < 0.05) (see Table 3).

### 3.4. Comparison of REE between the Two Groups before and after Surgery

Before operation, there was no significant difference in REE levels between the two groups (*P* > 0.05); the REE levels in the observation group were lower than those in the control group after 1, 2, and 3 days of operation, and the differences were statistically significant (*P* < 0.05) (see Table 4).

### 3.5. Comparison of T Cell Subset Levels between the Two Groups before and after Surgery

Before operation, there was no significant difference in serum CD3+, CD4+, and CD8+ levels between the two groups (*P* > 0.05); 3 days after operation, the serum CD3+ and CD4+ levels in the two groups were decreased, and the observation group was higher than the control group, and the difference was statistically significant (*P* < 0.05) (see Table 5).

### 3.6. Comparison of the Incidence of Complications between the Two Groups

The incidence of complications in the observation group (3.28%) was lower than that in the control group (13.11%), and the difference was statistically significant (*P* < 0.05) (see Table 6).

### 3.7. Comparison of Survival Time between Two Groups

There was no significant difference in the survival rate between the two groups at 1, 2, and 3 years of follow-up (*P* > 0.05) (see Table 7). The survival curve with follow-up of 1 to 3 years is shown in Figures 1–3.

RETRACTED

## 4. Discussion

Laparoscopic technology has been widely used in the treatment of colorectal cancer [11–13]. Compared with traditional open surgery, laparoscopic surgery has minimally invasive advantages such as less trauma, less postoperative pain, and faster recovery. However, there are still some shortcomings of laparoscopy, such as two-dimensional imaging, inflexible operation of instruments, and uncomfortable position of the operator, which limit the further application of laparoscopy in delicate surgery. Da Vinci robot-assisted surgery is a new type of surgery, which has certain advantages over traditional laparoscopic hepatectomy. This operation started late but developed rapidly, requiring nurses to have a high degree of surgical cooperation, and need to be equipped with a professional surgical team to deal with all kinds of unexpected situations. Surgical participants need to undergo strict and systematic robot operation training and master the correct operation and basic debugging of Da Vinci robot system. They need to complete various system inspections before the operation to ensure smooth operation. Leonardo's robot surgical system consists of three parts: doctor's console, bedside operating arm, and video screen system. Compared with traditional laparoscopic hepatectomy, the robotic surgical system has a clearer field of vision, and the 3D surgical field can be magnified 10 to 15 times, which is conducive to instrument operation and accurate positioning. The operation method is more precise, and it can perform delicate surgical operations in the space that cannot be touched by human hands, which overcomes some shortcomings of laparoscopic surgery. In addition, the mechanical arm is similar to and synchronized with the human hand, which is beneficial for doctors to quickly learn operations [14–16].

In this study, the observation group was treated with robot-assisted laparoscopic treatment, and the control group was treated with traditional laparoscopic treatment. The results showed that, after surgery, the operative time, intraoperative blood transfusion, intraoperative blood loss, and average intraoperative blood transfusion in the observation group were all less than those in the control group, indicating that robot-assisted laparoscopic therapy can effectively shorten the operative time and reduce intraoperative blood transfusion and intraoperative blood loss. At present, there are few clinical studies on robot-assisted laparoscopic hepatectomy, and it is speculated that the mechanism of shortening the operation time may be that the combined application of robot and laparoscopy can remove the lesion more quickly, the operation time is short, the trauma is small, and the intraoperative blood transfusion and blood loss of patients are significantly reduced.

RETRACTED

Stress response refers to a systemic nonspecific adaptive response caused by internal and external factors such as surgery and trauma. Cor, NE, and Glu are common stress indicators [17, 18]. Both robot-assisted laparoscopic hepatectomy and laparoscopic hepatectomy are traumatic operations, which can cause damage to the body tissue and lead to stress reaction. In this study, after 3 days of surgery, serum levels of Cor, NE, and Glu in the two groups increased, and the levels of Cor, NE, and Glu in the observation group were lower than those in the control group, indicating that the stress response index levels of the observation group changed little before and after surgery, and the stress response of the observation group was small. It is suggested that compared with traditional laparoscopic surgery, robot-assisted laparoscopic hepatectomy can effectively relieve patients' stress response, which may be because robot-assisted laparoscopic surgery is more delicate as a minimally invasive surgery and it can reduce the trauma to patient's body and relieve stress response. The body may be in a high metabolic state when it is injured, and REE is a common indicator for clinical evaluation of human metabolism [19, 20].

In this study, the REE levels of the two groups were higher after 1, 2, and 3 days of surgery than before surgery, indicating that both surgical methods caused trauma to the patient's body, resulting in a high metabolic state of the body. However, from 1 day after surgery, REE values of the observation group were lower than those of the control group, indicating that robot-assisted laparoscopic surgery has a slight impact on the body's energy metabolism, and patients' hypermetabolic state is easier to recover.

CD3+, CD4+, and CD8+ belong to T cell subsets. In this study, compared with the preoperative level, the levels of CD3+ and CD4+ in both groups decreased after surgery, indicating that there was immune damage in both groups. Three days after surgery, the levels of CD3+ and CD4+ in the observation group were higher than those in the control group, indicating that robot-assisted laparoscopy can effectively reduce immune injury and patients' postoperative immune function is easier to recover, which may be related to the effect of robot-assisted laparoscopy on reducing the body's stress response.

The incidence of complications in the observation group was lower than that in the control group. Compared with traditional laparoscopic surgery, robot-assisted laparoscopic surgery has more precise operation, wider field of view, more accurate positioning, and better surgical completion, so the incidence of complications such as incision infection, abdominal bleeding, pleural effusion, biliary leakage, and intestinal obstruction is significantly reduced.

RETRACTED

There was no significant difference in survival time between the two groups during 3-year follow-up, indicating that there was no significant difference in long-term prognosis between robot-assisted laparoscopic and traditional laparoscopic treatment for sCRLM. There have been no studies on the long-term prognosis of robot-assisted laparoscopic treatment for sCRLM in the past, and the specific conclusions need to be further explored.

In conclusion, robot-assisted laparoscopic treatment for sCRLM can effectively improve the perioperative situation of patients, relieve stress response, energy metabolism, and cellular immunity, and effectively reduce the occurrence of complications, which has clinical application value.

## Figures and Tables

**Figure 1:** Survival curve of 1-year follow-up.

**Figure 2:** Survival curve of 2-year follow-up.

**Figure 3:** Survival curve of 3-year follow-up.

**Table 1:** Comparison of baseline data between the two groups (*n* = 122).

Item	Observation group (*n* = 61)	Control group (*n* = 61)	*t/χ* ^2^ */*Fisher exact probability value	*P* value
Gender (*n* (%))				
Male	44 (72.13)	38 (62.30)	1.399	0.247
Female	17 (27.87)	23 (37.70)		
Age (years)	57.13 ± 5.86	57.51 ± 6.27	0.343	0.732
BMI	23.45 ± 2.32	23.59 ± 2.22	0.341	0.734
Site of the primary lesion (cases (%))				
Left colon	25 (40.98)	28 (45.90)	0.532	0.766
Right colon	6 (9.84)	7 (11.48)		
Rectum	30 (49.18)	26 (42.62)		
Differentiation degree				
Well differentiated	59 (96.72)	55 (90.16)	0.272	-
Poorly differentiated	2 (3.28)	6 (9.84)		
Maximum diameter of primary tumor (cm)	3.97 ± 1.44	4.05 ± 1.74	0.284	0.777
ASA score (cases (%))				
I~II	49 (80.33)	44 (72.13)	1.131	0.288
III	12 (19.67)	17 (27.87)		
Lymph node metastasis of the primary lesion (cases (%))				
Negative	21 (34.43)	17 (27.87)	0.612	0.434
Positive	40 (65.57)	44 (72.13)		
Depth of primary tumor invasion (cases (%))				
T1/T2	3 (4.92)	5 (8.20)	0.717	-
T3/T4	58 (95.08)	56 (91.80)		
Number of liver metastases (number)	2.10 ± 0.98	2.00 ± 1.20	0.497	0.620
Maximum diameter of liver metastases (cm)	2.91 ± 1.43	2.70 ± 1.35	0.829	0.409
Preoperative chemotherapy (cases (%))				
None	38 (62.30)	40 (65.57)	0.142	0.706
Yes	23 (37.70)	21 (34.43)		
Postoperative chemotherapy (cases (%))				
FOLFOX	36 (59.02)	40 (65.57)	0.772	-
XELOX	20 (32.79)	17 (27.87)		
Others	5 (8.20)	4 (6.56)		
Preoperative CEA (cases (%))				
≤5 *μ*g/l	18 (29.51)	21 (34.43)	0.339	0.560
>5 *μ*g/l	43 (70.49)	40 (65.57)		
Distribution of liver metastases (cases (%))				
Single lobe	40 (65.57)	37 (60.66)	0.317	0.573
Double lobes	21 (34.43)	24 (39.34)		

RETRACTED

**Table 2:** Comparison of perioperative conditions between the two groups (*x̅*±*s*).

Group	Operation time (min)	Intraoperative blood loss (ml)	Average intraoperative blood transfusion (ml)	Hepatic porta occlusion time (min)
Observation group (*n* = 61)	156.34 ± 15.97	203.11 ± 10.98	608.31 ± 117.08	39.39 ± 5.41
Control group (*n* = 61)	184.18 ± 18.03	356.00 ± 32.00	656.21 ± 103.75	40.52 ± 4.46
*t/χ* ^2^ value	9.027	35.123	2.392	1.260
*P* value	<0.001	<0.001	0.018	0.210

**Table 3:** Comparison of stress response index levels between the two groups before and after surgery (*x̅*±*s*).

Group	Cor (ng/ml)		NE (ng/l)		Glu (mmol/l)	
	Before surgery	3 days after surgery	Before surgery	3 days after surgery	Before surgery	3 days after surgery
Observation group (*n* = 61)	62.74 ± 5.86	72.65 ± 7.57^a^	157.11 ± 15.00	174.84 ± 16.30^a^	4.51 ± 0.44	5.74 ± 0.51^a^
Control group (*n* = 61)	62.41 ± 5.18	82.52 ± 7.11^a^	158.69 ± 16.79	190.22 ± 20.89^a^	4.53 ± 0.56	6.30 ± 0.61^a^
*t* value	0.663	5.915	0.553	4.535	0.170	5.464
*P* value	0.508	<0.001	0.581	<0.001	0.865	<0.001

Note: a represents *P* < 0.05 compared with the same group before surgery.

**Table 4:** Comparison of REE between the two groups before and after surgery (*x̅*±*s*, kj*/*d).

Group	Before surgery	1 day after surgery	2 days after surgery	3 days after surgery
Observation group (*n* = 61)	4432.97 ± 367.96	5114.69 ± 434.96^bcd^	5497.34 ± 384.70^cd^	4859.10 ± 400.44^d^
Control group (*n* = 61)	4455.58 ± 389.92	5895.01 ± 498.00^b^	6160.08 ± 587.51^b^	6473.75 ± 417.87^bc^
*t* value	0.329	9.217	7.371	21.789
*P* value	0.742	<0.001	<0.001	<0.001

Note: b represents *P* < 0.05 compared with before surgery; c represents *P* < 0.05 compared with 1 day after surgery; d represents *P* < 0.05 compared with 2 days after surgery.

**Table 5:** Comparison of T cell subset levels between the two groups before and after surgery (*x̅*±*s*, %).

Group	CD3+		CD4+		CD8+	
	Before surgery	3 days after surgery	Before surgery	3 days after surgery	Before surgery	3 days after surgery
Observation group (*n* = 61)	55.42 ± 5.35	49.89 ± 4.15^a^	31.48 ± 2.80	27.75 ± 2.41^a^	25.71 ± 2.43	26.81 ± 2.55^a^
Control group (*n* = 61)	55.08 ± 4.73	47.60 ± 4.06^a^	31.86 ± 2.92	25.30 ± 2.36^a^	25.48 ± 2.41	26.80 ± 2.80^a^
*t* value	0.772	3.072	0.744	5.880	0.527	0.013
*P* value	0.442	0.003	0.458	<0.001	0.599	0.990

Note: a represents *P* < 0.05 compared with the same group before surgery.

RETRACTED

**Table 6:** Comparison of the incidence of complications between the two groups (cases (%)).

Group	Incision infection	Abdominal hemorrhage	Pleural effusion	Bile leakage	Intestinal obstruction	Total complications
Observation group (*n* = 61)	0 (0.00)	0 (0.00)	1 (1.64)	0 (0.00)	1 (1.64)	2 (3.28)
Control group (*n* = 61)	1 (1.64)	1 (1.64)	2 (3.28)	2 (3.28)	2 (3.28)	8 (13.11)
*χ* ^2^ value						3.921
*P* value						0.048

**Table 7:** Comparison of survival time between two groups (cases (%)).

Group	1-year follow-up		2-year follow-up		3-year follow-up	
	Survival	Death	Survival	Death	Survival	Death
Observation group (*n* = 61)	52 (85.25)	9 (14.75)	43 (70.49)	18 (29.51)	31 (50.82)	30 (49.18)
Control group (*n* = 61)	48 (78.69)	13 (21.31)	40 (65.57)	21 (34.43)	26 (42.62)	yn (57.38)
Log-rank *χ*^2^ value	0.884		0.470		0.961	
*P* value	0.347		0.493		0.327	

## Data Availability

The labeled dataset used to support the findings of this study are available from the corresponding author upon request.
